# The Protective Effect of Artesunate on LPS-Induced Acute Respiratory Distress Syndrome through Inhibiting NLRP3 Inflammasome Signaling

**DOI:** 10.1155/2022/7655033

**Published:** 2022-08-23

**Authors:** Yifei Cui, Wenbo Weng, Qing Ding, Qinghua Su, Xiaoying Wang

**Affiliations:** ^1^Department of Pharmacy, The Children's Hospital, Zhejiang University School of Medicine, National Clinical Research Center for Child Health, Hangzhou, China; ^2^The Yuyao Health Further Education School, Ningbo, China; ^3^Department of Pediatrics, The First People's Hospital of Jiande, Hangzhou, China

## Abstract

**Background:**

Artesunate (AS) is a derivative of artemisinin that can exert anti-inflammatory effects. This study aims to explore the effect of AS on lipopolysaccharide (LPS)-induced acute respiratory distress syndrome (ARDS).

**Methods:**

The newborn mice were used for experimental ARDS model establishment by intraperitoneal injection of LPS (10 mg/kg) into mice with or without AS (20 mg/kg) pretreatment. After that, the pathological morphology of mouse lung tissue was observed by H&E staining. The content of inflammatory factors in serum was measured by ELISA and mRNA expression and lung tissue was determined by qRT-PCR. The expression of NLRP3 inflammasome and related proteins in lung tissue was confirmed by immunohistochemistry and Western blot.

**Results:**

AS treatment effectively alleviated the LPS-induced lung injury and pulmonary edema, and reduced the expression of IL-1*β*, IL-18, IL-6, IL-8, MCP-1, and TNF-*α* in serum and lung tissues of experimental ARDS mice. In addition, AS treatment reduced the expression of NLRP3, ASC, and caspase-1 in lung tissues of experimental ARDS mice.

**Conclusion:**

AS alleviated LPS-induced lung injury in ARDS mice by inhibiting the activation of NLRP3 inflammasome.

## 1. Introduction

Acute respiratory distress syndrome (ARDS) is an acute pulmonary inflammation syndrome characterized by diffuse inflammation of the lung parenchyma and the resulting osmotic pulmonary edema [1]. Taken together, severe pneumonia, sepsis, severe trauma, etc., are the main causes of ARDS [2]. Among them, ARDS caused by sepsis is very common in clinic, and its fatality rate is also higher than ARDS caused by other reasons [2, 3]. Moreover, the occurrence of ARDS in neonatus is more fatal, which is the most common problem in neonatal ICU and remains an important challenge for the intensive care clinician [4]. Studies have shown that the level of lipopolysaccharide (LPS) is closely related to the occurrence of ARDS caused by sepsis [5, 6]. Therefore, ARDS induced by LPS is a hot topic of current research and will be one of the focuses of this article. So far, the treatment of ARDS is still based on mechanical ventilation and nutritional support [7]. Although some drugs for the treatment of ARDS have been evaluated in clinical trials, the development of effective new drugs for the treatment of ARDS remains imminent [7, 8].

Natural products and their derivatives, such as baicalin, emodin, and resveratrol, have been successively reported to have great potential in the treatment of ARDS [9–11]. The mechanism of these substances in the treatment of ARDS is mainly related to the regulation of inflammatory response. Artesunate (AS) is a derivative of the antimalarial drug artemisinin. It is clinically used to treat malaria with good curative effects and low side effects [12]. In addition to the antimalarial effect, AS also has many pharmacological effects, such as immune regulation, anti-inflammation, antibacterial sensitization, anti-tumor, and so on [13]. Evidences also have suggested that AS acts as a good anti-inflammatory part in rheumatoid arthritis [14], ulcerative colitis [15], osteoarthritis [16], and other inflammatory disease models. However, whether AS improves LPS-induced ARDS by exerting anti-inflammatory effect is unclear.

NLRP3 inflammasome is one of the significant pathways regulating chronic inflammation, and it includes NLRP3, apoptosis-related speckle-like protein (ASC), and caspase-1 [17]. Zhang et al. found that melatonin can reduce acute lung injury by inhibiting the activation of NLRP3 inflammasomes [18]. Li et al. also found that pirfenidone improved LPS-induced ARDS by blocking the activation of NLRP3 [19]. It is worth noting that AS also can inhibit the pulmonary inflammation caused by renal ischemia-reperfusion via suppressing the activation of NLRP3 inflammasomes [20]. Therefore, we speculate that AS may improve the LPS-induced ARDS by regulating the NLRP3 inflammasomes. In this study, we established an experimental ARDS in newborn mice, to investigate whether AS could improve LPS-induced ARDS by exerting anti-inflammatory effect via NLRP3 inflammasomes, and the study confirms our conjecture.

## 2. Materials and Methods

### 2.1. Animals

40 C57BL/6 mice (male, 7 days) were purchased from Shanghai Lingchang Biotech Co., Ltd (SCXK 2018–0003). The mice were kept in an environment with a relative humidity of 22 ± 2°C. Animal experiments conducted in this study were approved by Animal Ethics Committee of Hangzhou Eyoung Biomedical Research and Development Center in accordance with the guidelines of the Institutional Animal Care and Use Committee.

The establishment of ARDS models was carried out according to the previous studies [21, 22]. A total number of 40 mice were randomly divided into 4 groups (control, LPS, LPS + AS, and AS), with 10 mice in each group. Mice in the LPS + AS and AS groups were intraperitoneally injected with 20 mg/kg of AS (SA9720, Solarbio, China), while mice in the LPS and control groups were intraperitoneally injected with the same amount of normal saline instead. Six hours after AS or saline injection, the mice in the LPS and LPS + AS groups were intraperitoneally injected with 10 mg/kg of LPS (L8880, Solarbio, China), while the mice in the control and AS groups were intraperitoneally injected with the same amount of saline. The slight tracheal rales from mice indicates successful ARDS model [23]. After 72 hours, the mice were euthanized and lung tissue and blood samples were collected.

### 2.2. Hematoxylin and Eosin (H&E) Staining

After the mouse lung tissue was fixed, it was embedded in paraffin and sectioned. After the paraffin sections are immersed in xylene and gradient alcohol, they are immersed in hematoxylin staining solution (E607317, Sangon, China) for 4 minutes. After washing, the slices are reacted with 1% hydrochloric acid alcohol and 0.6% ammonia water in turn, and then immersed in eosin dye solution (E607321, Sangon, China) for 5 minutes. Finally, the slices are dehydrated and mounted. A microscope (200× and 400 ×) was used to observe the results. The lung injury was scored according to the H&E staining scoring standards described previously [24].

### 2.3. Lung Wet Weight-to-Dry Weight Ratio Detection

After blotting the blood on the lung surface with filter paper, the wet weight of the lung was measured. The left lung was baked in an oven at 80°C for 48 hours until the weight remained unchanged, and then weighed. Lung W/D ratio = lung wet weight/lung dry weight.

### 2.4. Enzyme-Linked Immunosorbent Assay (ELISA)

The blood was centrifuged at 3500 r/min for 15 minutes to collect the supernatant. The levels of IL-1*β*, IL-18, IL-6, IL-8, MCP-1, and TNF-*α*in the serum were detected by the corresponding ELISA kit (MM-1011M2, MM-0123M2, MM-0040M2, MM-0122H2, MM-0169M2, MM-0082M2, MEIMIAN, China). In short, the antimouse antibody was coated on the enzyme plate in advance, and then the sample or standard was added to the enzyme plate to bind with the antibody, and the free components were washed away. Then biotinylated second antibody and horseradish peroxidase labeled avidin were added to the plate in turn. After washing away the free components, the enzyme plate was added with the chromogenic substrate for reaction. Finally, after adding the stop solution, detect the absorbance at 450 nm by a microplate reader (CMaxPlus, Molecular Devices, USA).

### 2.5. Quantitative Reverse Transcription Polymerase Chain Reaction (qRT-PCR) Assay

Total RNAs were collected from lung tissues by Trizol reagent (B511311, Sangon, China). Then cDNA was synthesized with the help of a reverse transcription kit (CW2569, CWBIO, China). QPCR was conducted in a real-time PCR system with the SYBR Premix Ex TaqII (RR820 A, Takara, Japan). Relative expressions were carried out using the 2^−ΔΔCt^ method. All the primer sequences were as follows (5′-3′). TNF-*α* : GCCACCACGCTCTTCTGTC, GCTACGGGCTTGTCACTCG; IL-1*β* : TTCAAATCTCACAGCAT, CACGGGCAAGACATAGGTAG; IL-6 : AACTCCATCTGCCCTTCA, CTGTTGTGGGTGGTATCCTC; GAPDH : AGGTCGGTGTGAACGGATTTG, GGGGTCGTTGATGGCAACA. GAPDH was used as the internal control.

### 2.6. Immunohistochemistry Assay

Paraffin sections were dewaxed and hydrated in xylene and gradient alcohol, and then heated in microwave oven for antigen repair. After that, the sections were incubated in 3% hydrogen peroxide solution for half an hour, and then sealed with 3% BSA (E661003, Sangon, China). After shaking off the blocking solution, the sections were reacted with anti-NLRP3 antibody (ab214185, ABCAM, UK) overnight at 4°C. After that, the sections were reacted with Goat Anti-Rabbit IgG (ab205718, ABCAM, China) at room temperature for 50 minutes. The color development of sections was completed by AEC Immunohistochemistry Color Development Kit (E670031, Sangon, China). The sections need to be re-dyed in hematoxylin solution for 3 minutes after color development. After sealing the sections, the results were observed under a microscope (magnification, 200× and 400 ×).

### 2.7. Western Blot Assay

RIPA buffer (R0010, Solarbio, China) was used to extract total protein. BCA Protein Assay Kit (PC0020, Solarbio, China) was then employed to quantify proteins in the lysates. Electrophoresis was then conducted to separate the proteins on nitrocellulose membranes. The blocking buffer (SW3015, Solarbio, China) was used block membrane. Then the membranes were reacted with antibodies. Antibodies were purchased from Affinity (USA) : IL-1*β* (1/1000, AF5103), ASC (1/1000, DF6304), NLRP3 (1/1000, DF7438), caspase-1 (1/1000, AF5418), IL-18 (1/1000, DF6252), p–NF–kB P65 (1/1000, AF5006), NF-kB P65 (1/1000, AF2006), TLR2 (1/1000, DF7002), TLR4 (1/5000, AF7017), *β*-actin (1/5000, AF7018), Rabbit IgG (1/5000, S0001). Finally, exposure was carried out by ECL chemiluminescent solution (36208ES60, Yeasen Biotech, China) on ChemiDoc MP Imager (BIO-RAD, USA).

### 2.8. Statistical Analyses

Graph Prism v8.0 (Graphpad software, California, USA) was employed to analyze the results. The data were represented as mean ± standard deviation. One-way analysis of variance was applied for the analysis of variance between multiple groups. *P* < 0.05 was considered statistically significant analysis.

## 3. Results

### 3.1. AS Reduced Lung Tissue Damages and W/D Ratio in LPS-Induced ARDS Mice

In LPS-induced ARDS mice, after AS treatment, the effect of AS on lung histopathologic changes was evaluated. As shown in Figure 1(a), the lung tissue structure in the control group was intact with no obvious abnormalities. However, in the H&E staining image of the LPS group, the alveolar hemorrhage, thickening of the alveolar septum, and inflammatory cell infiltration can be observed (*P* < 0.01). While these injuries were reduced in AS pre-treated group ARDS mice, accompanied with decreased HE score (*P* < 0.05). Furthermore, we also calculated the lung W/D ratio in each group mice. It could be observed that the induction of LPS increased the lung W/D ratio, caused pulmonary edema in ARDS mice, but it was reversed by the intervention of AS (Figure 1(b), *P* < 0.05).

### 3.2. AS Inhibited the Content of Inflammatory Factors in the Serum of ARDS Mice

In order to evaluate the anti-inflammation effect of AS on ARDS we detected the content of inflammatory factors in the serum by ELISA of ARDS mice. As shown in Figure 2, after LPS induction, the levels of IL-1*β*, IL-18, IL-6, IL-8, MCP-1, and TNF-*α* in the serum of ARDS mice increased sharply (*P* < 0.01). However, the treatment of AS can effectively inhibit the promoting effect of LPS on these inflammatory factors (*P* < 0.01).

### 3.3. AS Inhibited the mRNA Expression of TNF-*α*, IL-1*β,* and IL-6 in the Lung Tissues of ARDS Mice

The expression of inflammatory factors, including TNF-*α*, IL-1*β,* and IL-6, in the lung tissues were also detected by qRT-PCR assay. Consistent with the ELISA results, the mRNA levels of TNF-*α*, IL-1*β,* and IL-6 were elevated in LPS treated mice compared to the control group. While AS treatment significantly reversed the elevated mRNA expression levels of TNF-*α*, IL-1*β,* and IL-6 by LPS (Figure 3, *P* < 0.01).

### 3.4. AS Suppressed the NLRP3 Inflammasome Signaling in LPS-Induced ARDS Mice

The effect of AS on the NLRP3 inflammasome expression in LPS-induced ARDS mice was also investigated. The results of immunohistochemistry showed that the positive expression of the NLRP3 in the LPS group was higher than that in the control group (Figure 4). However, AS treatment suppressed the increase in NLRP3 expression caused by LPS.

Since NLRP3 forms NLRP3 inflammasomes with ASC and Caspase-1 to induce the release of IL-1*β* and IL-18, we also detected their expression in lung tissues. As shown in Figure 5, the protein expression levels of IL-1*β*, ASC, NLRP3, caspase-1, and IL-18 all significantly increased after LPS induction (*P* < 0.01), but in the AS intervention group, their protein levels all decreased to varying degrees (*P* < 0.05).

### 3.5. AS Suppressed the TLR4/NF-kB Pathway in LPS-Induced ARDS Mice

AS the TLR4/NF-kB pathway is critically involved in the inflammatory response, we further detect the expression of the proteins relevant to this pathway. As shown in Figure 6, the protein expressions of p–NF–kB P65, p–NF–kB P65/NF-kB P65, TLR2, and TLR4 were significantly activated in LPS group lung tissues (*P* < 0.01). While in LPS + AS treated group, the expressions of these proteins were suppressed by AS (*P* < 0.05).

## 4. Discussion

Previous studies have proved that AS can alleviate LPS-induced acute lung injury, which contributed to the regulation of inflammatory signaling, including TLR2, and Nrf2 [21, 25]. In this study, we focused on the anti-inflammatory effect of AS on ARDS. Our research has given a new clue of AS for the treatment of LPS-induced ARDS, which is by inhibiting the activation of NLRP3 inflammasome signaling to alleviate inflammatory injury of ARDS.

Studies have shown that inflammatory response is an important cause of ARDS, and blocking the progression of inflammatory response can effectively reduce the pathological injuries and symptom of ARDS [26, 27]. When the patient is in the early stage of the disease, the mononuclear-macrophage system in the body is activated, releasing IL-1*β*, IL-8, TNF-*α*, and other inflammatory factors. The interaction between these inflammatory factors promoted the production of chemokines, recruited inflammatory cells to infiltrate, triggered a cascade of inflammatory reactions, and ultimately led to lung tissue damage [27, 28]. Evidences have suggested that in the occurrence and development of ARDS, TNF-*α* and IL-1*β* can stimulate stromal cells and endothelial cells to produce chemokine MCP-1 in the inflammatory site, promote the infiltration of neutrophils and endothelial cells [28–30]. The reason why AS is used as an anti-inflammatory drug for inflammatory diseases contributes to its inhibition on the secretion of inflammatory factors and chemokines. Jiang et al. found that AS alone or in combination with rosuvastatin can inhibit the contents of TNF-*α*, IL-6, IL-6, and MCP-1, thereby slowing the development of atherosclerosis [31]. Cao et al. found that AS can reduce TNF-*α* and IL-6 contents in serum and bronchoalveolar lavage fluid (BALF) of mice with septic lung injury [32]. Similarly, in our study, AS inhibited the secretion of inflammatory factors, including IL-1*β*, IL-18, IL-6, IL-8, MCP-1, and TNF-*α* in serum and lung tissues, alleviated lung tissue damages, and pulmonary edema in model mice. These fundings indicated that AS could suppressed the LPS-induced inflammation and lung injury, thus showing a therapeutic effect on LPS-induced ARDS.

NLRP3 inflammasome participates in the body's immune defense, but excessive activation can cause inflammation-related damage. The activation of NLRP3 can cause the aggregation of ASC, which in turn leads to the cleavage of pro-caspase-1 into caspase-1, and ultimately promotes the mature secretion of downstream inflammatory factors, thereby inducing chronic inflammation in the body. It is reported that the NLRP3 inflammasome could be activated in the LPS-induced ARDS model in mice [33]. A similar phenomenon was also observed in mouse model in our study. However, by inhibiting the activation of NLRP3 inflammasome, it can well reduce the severity of ALI in experimental mice [33]. NLRP3 is not only involved in LPS-induced ALI, but also in ARDS caused by mechanical ventilation, COPD, and other chronic lung diseases [34, 35]. Jones et al. constructed ARDS mice model through the dual effects of mechanical ventilation and LPS, and found that the level of IL-1*β* in the BALF of ARDS mice with NLRP3 deficiency and caspase-1 ischemia was significantly reduced, and hypoxia was also alleviated [34]. These evidences suggest that ARDS can be improved by preventing excessive activation of NLRP3 inflammasomes. In our study, the activation of NLRP3 inflammasome in LPS-induced ARDS mice was inhibited by AS intervention treatment, accompanied with the reduced lung injury and inflammation, indicating that AS may be a candidate drug for LPS-induced ARDS.

All the same, our research also has shortcomings. We only verified the regulatory effect of AS on the downstream products of NLRP3 inflammasome activation, but did not study the upstream link of NLRP3 inflammasome activation. Further in-depth study is needed to clarify the clear role of AS in ARDS.

In general, our study proved that AS alleviated LPS-induced lung injury in ARDS mice by inhibiting the activation of NLRP3 inflammasome and provided a new theoretical basis for AS treatment of ARDS.

## Figures and Tables

**Figure 1:** Effect of AS on pathological changes of lung tissue in LPS-induced experimental ARDS mice. Newborn mice were treated with AS and LPS successively, then lung tissues were obtained for pathological analysis.(a) H&E staining of lung tissue, magnification: 200× and 400×.(b) Lung wet weight-to-dry weight ratio. ^▲▲^*P* < 0.01 vs. Control group; ^★^*P* < 0.05 vs. LPS group. AS: artesunate. LPS : Lipopolysaccharide.

**Figure 2:** Effect of AS on the contents of inflammatory factors in the serum of LPS-induced ARDS mice. The contents of IL-1*β*, IL-18, IL-6, IL-8, MCP-1, and TNF-*α* in serum were detected by ELISA. ^▲▲^*P* < 0.01 vs. Control group. ^★★^*P* < 0.01 vs. LPS group. AS: artesunate. LPS : Lipopolysaccharide.

**Figure 3:** Effect of AS on the contents of inflammatory factors in the lung tissues of LPS-induced ARDS mice. The relative expression levels of TNF-*α*, IL-1*β,* and IL-6 in the lung tissues of each group of mice were determined by qRT-PCR. ^▲▲^*P* < 0.01 vs. Control group. ^★★^*P* < 0.01 vs. LPS group. AS: artesunate. LPS : Lipopolysaccharide.

**Figure 4:** The effect of AS on the NLRP3 inflammasome expression in LPS-induced ARDS mice. The positive expression of NLRP3 in the lung tissues of each group of mice were determined by immunohistochemistry, magnification: 200× and 400×. AS: artesunate. LPS : Lipopolysaccharide.

**Figure 5:** The effect of AS on the NLRP3 inflammasome signaling pathway related proteins expression in LPS-induced ARDS mice. Western blot was used to detect the relative protein expression of NLRP3, ASC, Caspase-1, IL-18, and IL-1*β* in the lung tissue of each group of mice, *β*-actin was used as the internal control. ^▲▲^*P* < 0.01 vs. Control group. ^★^*P* < 0.05 vs. LPS group. AS: artesunate. LPS : Lipopolysaccharide.

**Figure 6:** The effect of AS on the TLR4/NF-kB pathway related proteins expression in LPS-induced ARDS mice. Western blot was used to detect the relative protein expression of p–NF–kB P65, NF-kB P65, TLR2, and TLR4 in the lung tissue of each group of mice, *β*-actin was used as the internal control. ^▲▲^*P* < 0.01 vs. Control group. ^★^*P* < 0.05 vs. LPS group. AS: artesunate. LPS : Lipopolysaccharide.

## Data Availability

The data used to support the findings of this study are available from the corresponding author upon request.
